RETRACTED

# The Diagnostic Accuracy of Transabdominal and Transvaginal Color Doppler Ultrasound for Pregnant Women with Vasa Previa and Velamentous Cord Insertion

**DOI:** 10.1155/2022/1685783

**Published:** 2022-09-29

**Authors:** Qing Liu, Qiang Zhang, Peiwu Liu

**Affiliations:** ^1^Department of Ultrasound, Jingzhou Hospital Affiliated to Yangtze University, China; ^2^Radiology Department, Jingzhou Hospital Affiliated to Yangtze University, China

## Abstract

**Objective:**

The objective of this study is to evaluate feasibility and accuracy of transabdominal color Doppler ultrasound (TA-CDUS) and transvaginal color Doppler ultrasound (TV-CDUS) as screening methods for pregnant women with vasa previa (VP) and velamentous cord insertion (VCI).

**Methods:**

A retrospective diagnostic accuracy study was performed on 5,434 pregnant women from 2018 to 2021, who underwent both TA-CDUS and TV-CDUS. Diagnostic performance of TA-CDUS and TV-CDUS was determined using specificity, positive predictive value (PPV), negative predictive value (NPV), accuracy, and positive and negative likelihood ratios (LR^+^ and LR^−^), using the delivery information (gross examination) as the “Gold-standard”. Patient records were reviewed for demographics and diagnosis.

**Results:**

The combination of VP and VCI was diagnosed in 37/5434 (0.68%) women at delivery. The sensitivity, specificity, PPV, NPV, and overall test accuracy of TA-CDUS were 72.97%, 99.85%, 77.14%, 99.81%, and 99.67%, respectively, for diagnosing VP with VCI. The corresponding values for TV-CDUS were 89.19%, 99.87%, 82.50%, 99.93%, and 99.80%, respectively. Moreover, the sensitivity of combination of TA-CDUS and TA-CDUS in determining VP with VCI was 97.30%, specificity 99.98%, PPV 97.30%, NPV 99.98%, and accuracy 99.96%. No significant difference in the misdiagnosis and missed diagnosis was found between the examination by TA-CDUS and TV-CDUS.

**Conclusions:**

Both TA-CDUS and TV-CDUS can be acceptable diagnostic tools for assessment of pregnant women with VP and VCI, with a better application of TV-CDUS with higher accuracy. The combination of TA-CDUS and TV-CDUS could provide an objective imaging basis for choosing clinical treatment strategies and predicting prognosis.

## 1. Introduction

Vasa previa (VP) are the umbilical vessels that is a complication of pregnancy in which fetal blood vessels lie outside the chorionic plate, in close proximity to the internal cervical os [1], which has been usually classified into (1) vessels connect a velamentous cord insertion (VCI) to the placenta and (2) vessels connect the lobes of a bilobed placenta or the placenta to a succenturiate lobe [2]. In VP cases, the protection of the umbilical cord by placental tissue or Wharton's jelly is absent, and the compression of the umbilical vessels may result in fetal heart decelerations and blood loss, as well as fetal mortality [3, 4]. It was reported that VP has an incidence of 0.0004~0.08% with a high fetal mortality due to fetal exsanguination [5, 6], which was commonly caused by second trimester low-lying placenta/placenta previa, bilobed/succenturiate lobe placenta, assisted reproductive technologies, vaginal bleeding, multiple gestation, and first trimester umbilical cord insertion in the lower 1/3 of the uterus [7].

RETRACTED

VCI as a rare placental abnormality had an incidence of 0.23~1% and 15% in singleton gestation and monochorionic twin pregnancies, respectively [8, 9]. The associated pathology for VP is mainly fetal heart abnormalities, and the risk factors are assisted reproduction, low-lying placenta, placenta previa, accessory lobe/bilobated placenta, and multiple pregnancy [6]. VP prenatally with VCI may be associated with several pregnancy outcomes, such as preterm delivery and postpartum hemorrhage [6, 10, 11]. The antenatal diagnosis increases the neonatal survival from 44% to 97% and improves the neonatal outcome [12]. Therefore, the correct diagnosis of the general classification of umbilical cord anomalies, namely, VP and VCI, is clinically important, while it still remains a challenge recently in the obstetrical practice.

Color Doppler ultrasound is a noninvasive diagnostic method for clinical diagnosis of obstetrics and gynecology diseases, which can be used to detect blood flow signals and highlight the umbilical vessel pathway [9, 13], which have proven to be valuable antepartum diagnostic tools for the early recognition of VP [14]. Moreover, ultrasound used color Doppler had a 74.1% sensitivity for the diagnosis of VCI with a positive predictive value (PPV) of 90.9% [15, 16], which was reported to have increased sensitivity to 100% with a lower PPV (85.7%) after the limited analysis by Rodriguez D et al. [17]. Currently, transabdominal color Doppler ultrasonography (TA-CDUS) and transvaginal color Doppler ultrasonography (TV-CDUS) are both used in the clinical diagnosis of several diseases, such as uterine adenomyoma and uterine fibroids [18], endometrial polyps [19], and ventriculo-coronary communications [20]. However, both of which have their own advantages and limitations [18]. Transabdominal ultrasound (TAS) and transvaginal ultrasound (TVS) examinations performed during the mid-trimester are a valuable tool in terms of achieving a timely and accurate diagnosis of VP [21] or VCI [22], especially with the color Doppler, which could increase its diagnostic accuracy [19].

RETRACTED

At present, we determined the value and the comparison of TA-CDUS and TV-CDUS in distinguishing the patients with VP and VCI. Moreover, we also showed the combined value in the diagnosis of the included pregnant women.

## 2. Methods and Materials

### 2.1. Participants

We retrospectively reviewed the clinical data of 5,434 women from 2018 to 2021, who received cesarean delivery in our hospital. All participants at 22~36 weeks' gestation underwent both TA-CDUS and TV-CDUS Doppler ultrasound. Inclusion criteria are as follows: (1) older than 18 years and (2) of singleton pregnancy. Exclusion criteria are as follows: (1) patients with coagulation dysfunction; (2) women with incomplete data; (3) women with multiple pregnancies; and (4) patients were complicated with reproductive system malignancies.

### 2.2. Ultrasound Examinations with TA-CDUS and TV-CDUS

All patients were allotted approximately 20 min for TA-CDUS in the second trimester and TV-CDUS in the third trimester using Mindray Resona 7 (Shenzhen, China) and Voluson E10 GE ultrasound machine with an RM6C transducer (GE Medical Systems, Zipf, Austria) equipped with a transabdominal 1~5 MHz convex probe and with a 5~9 MHz convex vaginal transducer. After the bladder was emptied, the patient lays on the gynecologic examination table in the lithotomy position for TV-CDUS examination. After the coupling agent was applied on the surface of the probe, which was slowly sent to the vagina of the subject followed by placing in the external cervical opening of the vagina, for TA-CDUS examination, the patient was in a supine position on full bladder. A coupling agent was applied to the lower abdomen of the patient. The examiners were obstetricians/gynecologists, who had 3 to 5 years of experience.

### 2.3. Diagnostic Criteria for VP and VCI

The diagnosis of VP was made when the umbilical vessels located 2 cm proximal to the cervical os. The VCI was diagnosed by (1) umbilical vessels entering the placenta margin parallel to the uterine wall and connecting to superficial placental vessels; (2) the cord insertion was immobile, even when the uterus was shaken; and (3) the umbilical vessels diverged as they traversed the membrane. The representative image of patients with VP and VCI is illustrated in Figure 1.

### 2.4. Observation Index

Taking the delivery information (Figure 2) as the gold standard, the number of true positives, false positives, true negatives, and false negatives was determined and presented in a 2 × 2 contingency table. The diagnostic efficacy of TA-CDUS, TV-CDUS, and these combinations was compared by sensitivity, specificity, positive predictive value (PPV), negative predictive value (NPV), and accuracy, as well as the positive and negative likelihood ratios (LR^+^ and LR^−^).

RETRACTED

### 2.5. Statistical Analysis

The sample is described in its clinical and demographic characteristics using quantitative variables, which are summarized with mean and standard deviation (SD). The categorical data of misdiagnosis and missed diagnosis using TA-CDUS and TV-CDUS are expressed as frequencies and percentages, which were evaluated and compared using *χ*^2^ test in SPSS 22.0 software for Windows (SPSS Inc., Chicago, IL, USA). The data were considered no statistically significant at two-sided *P* ≥ 0.05.

## 3. Result

### 3.1. Patient Demographics

A total of 37 patients (0.68%) of 5434 pregnant mothers at delivery were clinically extraordinarily positive as VP prenatally with VCI and 5,397 patients (99.32%) were negative. The identification using TA-CDUS and TV-CDUS showed a total of 35 and 40 patients combined with VP and VCI, respectively. The demographics findings in 51 cases who were diagnosed as VP with VCI by delivery information, TA-CDUS, or TV-CDUS are shown in Table 1. The maternal age of participants was 28.65 (SD = 4.86) years with the body mass index (BMI) of 23.84 ± 3.54 kg/m^2^. The gravidity and parity of women were 2.59 ± 1.08 (range =1~5) and 0.65 ± 0.59 (range =0~2), respectively, with the gestational age at delivery of 35.43 ± 1.15 weeks and neonatal birth weight of 2653.86 ± 233.71 g. Moreover, smoking during pregnancy (>5 cigarettes/day) was seen in 3 (5.88%) cases. No pregnant woman had alcohol consumption during pregnancy.

### 3.2. Diagnostic Accuracy of TA-CDUS and TV-CDUS in Pregnant Women with VP and VCI

In order to show the diagnostic accuracy of TA-CDUS and TV-CDUS in pregnant women with VP and VCI, we used delivery information as the gold standard. As demonstrated in Table 2 and Figure 3(a), the LR^+^ is 492.29, and the LR^−^ is 0.27 by TA-CDUS diagnosis, with an overall sensitivity of 72.97%, specificity of 99.85%, PPV of 77.14%, NPV of 99.81%, and accuracy value of 99.67%. Furthermore, TV-CDUS showed a total of 40 positive patients and 5,394 negative ones, which indicated a sensitivity, specificity, PPV, NPV, and accuracy of 89.19%, 99.87%, 82.50%, 99.93%, and 99.80% (Figure 3(b)), respectively, for categorization of a patient with VP and VCI, with the LR^+^ of 687.65 and LR^−^ of 0.11 (Table 3).

### 3.3. Combining Diagnostic Value Using TA-CDUS and TV-CDUS

Diagnosis can be established by combining several sonographic measurements [23], and several researchers recommend using TA-CDUS in combination with TA-CDUS [18, 24]. As shown in Figure 3(c) and Table 4, the combined use of TA-CDUS and TV-CDUS produces a high sensitivity of 97.30%, specificity of 99.98%, PPV of 97.30%, NPV of 99.97%, and accuracy of 99.96% as well as a positive and negative LR of 5,251.14 and 0.03, respectively.

RETRACTED

### 3.4. Comparison of Misdiagnosis and Missed Diagnosis Using TA-CDUS and TV-CDUS

Ultrasound like any other radiological methods also has its limitations due to the misdiagnosis and missed diagnosis. According to the result of TA-CDUS, a total of 9 patients (0.17%) showed the missed diagnosis of VCI (*n* = 8) or VP (*n* = 1). Moreover, placenta previa with VP (*n* = 7) was the most common misdiagnosis, and the others causes for misdiagnosis were 1 patient with low-lying placenta + placental adhesions + lobulated placenta and 1 patient with low-lying placenta and VP. Additionally, 0.07% (4/5434) and 0.13% (7/5434) patients were missed and misdiagnosed based on the TV-CDUS. In detail, 3 cases and 1 case were missed diagnosed, who appeared to be only VCI or VP at delivery, respectively. Moreover, 7 patients were confirmed as placenta previa + VP (*n* = 4), VP + low-lying placenta + bilobed placenta (*n* = 1), VP + placental adhesions (*n* = 1), and VP + lobulated placenta (*n* = 1) based on the delivery information, who were all misdiagnosed as VP + VCI by TV-CDUS. No significant difference in the misdiagnosis (*P* = 0.165) and missed diagnosis (*P* = 0.617) was found between the examination by TA-CDUS and TV-CDUS.

## 4. Discussion

As the most useful modalities for imaging adult female genital organs, both TAS and TVS have been wildly used in antenatal ultrasound examination at home and abroad with superior spatial resolution, lack of ionizing radiation, and ability to assess blood flow [25–27]. Moreover, the improved sonographic assessment of the vascularity and blood flow within the uterus (both gravid and nongravid), fetus, and placenta using color Doppler has resulted in enhanced depiction of certain obstetric and gynecologic disorder [28].

Prenatal recognitions of VP and VCI provide elective delivery, thus avoiding potential fetal demise and neonatal morbidity [8, 29]. However, an increase in missed cases of VP is usually seen when the ultrasound examination does not involve color Doppler [1]. In our study, a total of 37 patients (0.68%) of 5434 pregnant mothers at delivery were clinically extraordinarily positive as VP prenatally with VCI, and the figure was similar with previous studies [30, 31]. The identification using TA-CDUS showed a total of 35 patients having VP with VCI, and taking the delivery information as “gold-standard,” the overall sensitivity of TA-CDUS was 72.97%, specificity 99.85%, PPV 77.14%, NPV 99.81%, and accuracy 99.67% accompanying by a total of 9 patients with missed diagnosis of VCI (*n* = 8) or VP (*n* = 1). Moreover, placenta previa with VP (*n* = 7) was the most common misdiagnosis in our analysis, and the other causes for misdiagnosis were 1 patient with low-lying placenta + placental adhesions + lobulated placenta and 1 patient with low-lying placenta and VP.

RETRACTED

In a study by S Baulies et al., which was performed on 9 patients to detect VP at 20~22 weeks, the findings of TV-CDUS were 100% of accuracy [32]. A retrospective study between 2006 and 2009 by Hasegawa J *et al.* showed that the diagnostic accuracy was 100% with TV-CDUS at second trimester [33]. The advantages of TVS over TAS have been well documented. For example, Mathis J *et al.* examined that the diagnostic performance of TVS was better than TAS for high-quality imaging of the uterus and the bilateral adnexa with a higher sensitivity and specificity [23]. Furthermore, TVS was considered superior in 63%, equal in 27%, and inferior in 10% of the cases as compared to TAS in the evaluation of pelvic pathology [34]. The results of this study showed that TV-CDUS had a sensitivity, specificity, PPV, NPV, and accuracy of 89.19%, 99.87%, 82.50%, 99.93%, and 99.80%, respectively, for categorization of a patient with VP and VCI. However, 3 cases and 1 case were missed diagnosed that appeared to be only VCI and VP at delivery, respectively. Moreover, 7 patients were confirmed as placenta previa + VP, VP + low-lying placenta + bilobed placenta, VP + placental adhesions, and VP + lobulated placenta based on the delivery information, who were all misdiagnosed as VP + VCI by TV-CDUS. All mentioned above indicated the higher diagnostic performance of TV-CDUS than TA-CDUS.

TVS as the procedure of choice in the evaluation of patients who have a suspected ectopic pregnancy is used as an adjunctive tool to complement TAS [35], and this combination is superior in imaging the placental type, location, insertion of the cord, and VP [36]. A prospective study by Nomiyama et al. focused on the detection of VCI and VP as primary objectives, and the result showed that the identification of a VCI site by ultrasound evaluation (TA-CDUS; TV-CDUS if cord insertion not seen in third trimester) had a sensitivity of 100%, a specificity of 99.8%, a PPV of 83%, and a NPV of 100% [15]. Furthermore, in a study by Catanzarite *et al.* which combined the TA-CDUS and TV-CDUS in the diagnosis of VP and VCI, reported 10 cases were confirmed at delivery, while the 11th case was a false-positive diagnosis that appeared to be a placenta previa with the specificity of 100% [37]. At present, the combined use of TA-CDUS and TV-CDUS produced a high sensitivity of 97.30%, specificity of 99.98%, PPV of 97.30%, NPV of 99.98%, and accuracy value of 99.96%, indicating the importance role of this combination in antenatal ultrasound examination. The main limitation of the study was the retrospective nature of the study design. A prospective study using these two scans for pregnant women is the next step to be undertaken. Moreover, although highly visualization of VCI combined with VP using TA-CDUS/TV-CDUS imaging was found in this analysis, ultrasound like any other radiological methods also has its limitations due to the misdiagnosis and missed diagnosis.

RETRACTED

## 5. Conclusion

TV-CDUS demonstrated higher diagnostic performance than TA-CDUS in pregnant women with VP and VCI, and these combinations are superior to TA-CDUS or TV-CDUS alone. The visualization of VCI combined with VP using TA-CDUS/TV-CDUS imaging is recommended as a routine part of obstetric sonography, since the identification of VCI, especially in the case of VP, could help to determine the mode and timing of delivery and improve fetal outcome.

## Figures and Tables

**Figure 1:** Color Doppler ultrasonography indicated the patients with VP + VCI (gestational week: 34+ 4 weeks; age: 31 years). Note: (a) TA-CDUS: the placenta was located on the posterior wall of the uterus near the internal os. (b) TV-CDUS: The umbilical vessel was fixed at the internal os with the adherence of the placenta to the posterior region. (c) The Doppler spectrum of the blood vessels above the internal os was consistent with the umbilical artery spectrum.

**Figure 2:** Gross placental specimen (normal placenta and vasa previa).

**Figure 3:** Sensitivity, specificity, PPV, NPV, and accuracy for the detection of patients with VP and VCI. Note: (a) TA-CDUS; (b) TV-CDUS; and (c) the combined use of TA-CDUS and TV-CDUS.

**Table 1:** The demographics findings in 51 cases who were diagnosed as VP with VCI using delivery information, TA-CDUS, or TV-CDUS.

	Mean ± SD	Range
Age (years)	28.65 ± 4.87	20~44
Gravidity	2.59 ± 1.08	1~5
Parity	0.65 ± 0.59	0~2
Gestational age at delivery (weeks)	35.43 ± 1.15	34~37
Body mass index (BMI, kg/m^2)^	23.84 ± 3.54	18.9~29.9
Neonatal birth weight (g)	2653.86 ± 233.71	2300~2999

**Table 2:** Positive and negative likelihood ratios (LR^+^ and LR^−^) of TA-CDUS examination in determining VP combined with VCI taking gross examination as the gold standard.

TA-CDUS	Gold standard			LR^+^	LR^−^
	Positive	Negative	Total		
Positive	27 (0.50%)	8 (0.15%)	35 (0.65%)	492.29	0.27
Negative	10 (0.18%)	5389 (99.17%)	5399 (99.35%)		
Total	37 (0.68%)	5397 (99.32%)			

**Table 3:** Positive and negative likelihood ratios (LR^+^ and LR^−^) of TV-CDUS examination in determining VP combined with VCI taking gross examination as the gold standard.

TV-CDUS	Gold standard			LR^+^	LR^−^
	Positive	Negative	Total		
Positive	33 (0.61%)	7 (0.13%)	40 (0.74%)	687.65	0.11
Negative	4 (0.07%)	5390 (99.19%)	5394 (99.26%)		
Total	37 (0.68%)	5397 (99.32%)			

RETRACTED

**Table 4:** Positive and negative likelihood ratios (LR^+^ and LR^−^) of combining diagnosis using TA-CDUS and TV-CDUS in determining VP plus VCI taking gross examination as the gold standard.

TA-CDUS + TV-CDUS	Gold standard			LR^+^	LR^−^
	Positive	Negative	Total		
Positive	36 (0.66%)	1 (0.02%)	37 (0.68%)	5251.14	0.03
Negative	1 (0.02%)	5396 (99.30%)	5397 (99.32%)		
Total	37 (0.68%)	5397 (99.32%)			

## Data Availability

The data were presented in the study.

## References

[1] Ruiter L., Kok N., Limpens J. (2015). Systematic review of accuracy of ultrasound in the diagnosis of vasa previa. *Ultrasound in Obstetrics & Gynecology*.

[2] Kamijo K., Miyamoto T., Ando H. (2021). Clinical characteristics of a novel “Type 3” vasa previa: case series at a single center. *Journal of Maternal-Fetal & Neonatal Medicine*.

[3] Gross A., Markota Ajd B., Specht C., Scheier M. (2021). Systematic screening for vasa previa at the 20-week anomaly scan. *Acta Obstetricia et Gynecologica Scandinavica*.

[4] Baumfeld Y., Gutvirtz G., Shoham I., Sheiner E. (2016). Fetal heart rate patterns of pregnancies with vasa previa and velamentous cord insertion. *Archives of Gynecology and Obstetrics*.

[5] Park J. N., Kim Y. H., Kim C. H. (2008). One case of prenatally diagnosed vasa previa accompanied by succenturiate placenta. *Korean Journal of Obstetrics and Gynecology*.

[6] Bohiltea R. E., Dima V., Ducu I. (2022). Clinically relevant prenatal ultrasound diagnosis of umbilical cord pathology. *Diagnostics (Basel)*.

[7] Sutera M., Garofalo A., Pilloni E. (2021). Vasa previa: when antenatal diagnosis can change fetal prognosis. *Journal of Perinatal Medicine*.

[8] Schoenen S., Emonts P., Van Linthout C. (2020). Velamentous cord insertion associated with vasa praevia. *Revue Medicale de Liege*.

[9] Bohiltea R. E., Cirstoiu M. M., Ciuvica A. I. (2016). Velamentous insertion of umbilical cord with vasa praevia: case series and literature review. *Journal of Medicine and Life*.

[10] Yerlikaya G., Pils S., Springer S., Chalubinski K., Ott J. (2016). Velamentous cord insertion as a risk factor for obstetric outcome: a retrospective case-control study. *Archives of Gynecology and Obstetrics*.

[11] Matsuzaki S., Ueda Y., Matsuzaki S. (2022). Assisted reproductive technique and abnormal cord insertion: a systematic review and meta-analysis. *Biomedicines*.

[12] Ruiter L., Kok N., Limpens J. (2016). Incidence of and risk indicators for vasa praevia: a systematic review. *BJOG: An International Journal of Obstetrics & Gynaecology*.

RETRACTED

[13] Zheng X., Li X., Xu J., Wei Y. (2021). Intelligent recognition algorithm-based color doppler ultrasound in the treatment of dangerous placenta previa. *Journal of Healthcare Engineering*.

[14] Fleming A. D., Johnson C., Targy M. (1996). Diagnosis of vasa previa with ultrasound and color flow doppler: a case report. *The Nebraska Medical Journal*.

[15] Nomiyama M., Toyota Y., Kawano H. (1998). Antenatal diagnosis of velamentous umbilical cord insertion and vasa previa with color doppler imaging. *Ultrasound in Obstetrics and Gynecology*.

[16] Sepulveda W., Rojas I., Robert J. A., Schnapp C., Alcalde J. L. (2003). Prenatal detection of velamentous insertion of the umbilical cord: a prospective color doppler ultrasound study. *Ultrasound in Obstetrics & Gynecology*.

[17] Rodriguez D., Eliner Y. (2019). Performance of ultrasound for the visualization of the placental cord insertion. *Current Opinion in Obstetrics and Gynecology*.

[18] Qi H., Zhou C., Huang Z., Yang N., Wu Q. (2022). Value of transabdominal combined transvaginal color doppler ultrasonography in the distinguish between uterine adenomyoma and uterine fibroids. *BioMed Research International*.

[19] Raz N., Feinmesser L., Moore O., Haimovich S. (2021). Endometrial polyps: diagnosis and treatment options - a review of literature. *Minimally Invasive Therapy & Allied Technologies*.

[20] Chaoui R., Tennstedt C., Goldner B., Bollmann R. (1997). Prenatal diagnosis of ventriculo-coronary communications in a second-trimester fetus using transvaginal and transabdominal color doppler sonography. *Ultrasound in Obstetrics and Gynecology*.

[21] Santos Roca A. J., Mejias Ramos J. L., Lynch L., De la Vega A. (2021). Prenatal diagnosis of vasa previa by routine transvaginal color doppler. *Puerto Rico Health Sciences Journal*.

[22] Hasegawa J., Matsuoka R., Ichizuka K. (2006). Cord insertion into the lower third of the uterus in the first trimester is associated with placental and umbilical cord abnormalities. *Ultrasound in Obstetrics and Gynecology*.

[23] Mathis J., Dong Y., Abendstein B. (2022). Normative values of the internal genital organs of the female pelvis in transvaginal and transabdominal ultrasound. *Medical Ultrasonography*.

[24] Andolf E., Jorgensen C. (1990). A prospective comparison of transabdominal and transvaginal ultrasound with surgical findings in gynecologic disease. *Journal of Ultrasound in Medicine*.

[25] Di Pasquo E., Volpe N., Labadini C. (2021). Antepartum evaluation of the obstetric conjugate at transabdominal 2D ultrasound: a feasibility study. *Acta Obstetricia et Gynecologica Scandinavica*.

RETRACTED

[26] Garofalo A., Pilloni E., Alemanno M. G. (2019). Ultrasound accuracy in prenatal diagnosis of abnormal placentation of posterior placenta previa. *European Journal of Obstetrics & Gynecology and Reproductive Biology*.

[27] Pilloni E., Alemanno M. G., Gaglioti P. (2016). Accuracy of ultrasound in antenatal diagnosis of placental attachment disorders. *Ultrasound in Obstetrics & Gynecology*.

[28] Fleischer A. C., Andreotti R. F. (2005). Color doppler sonography in obstetrics and gynecology. *Expert Review of Medical Devices*.

[29] Matsubara S., Kuwata T., Takahashi H., Suzuki H. (2016). Vasa previa: another ultrasound sign and caution at cesarean section. *The Journal of Maternal-Fetal & Neonatal Medicine*.

[30] Yang M., Zheng Y., Li M. (2020). Clinical features of velamentous umbilical cord insertion and vasa previa: a retrospective analysis based on 501 cases. *Medicine (Baltimore)*.

[31] Sherer D. M., Al-Haddad S., Cheng R., Dalloul M. (2021). Current perspectives of prenatal sonography of umbilical cord morphology. *International Journal of Women's Health*.

[32] Baulies S., Maiz N., Munoz A., Torrents M., Echevarria M., Serra B. (2007). Prenatal ultrasound diagnosis of vasa praevia and analysis of risk factors. *Prenatal Diagnosis*.

[33] Hasegawa J., Farina A., Nakamura M. (2010). Analysis of the ultrasonographic findings predictive of vasa previa. *Prenatal Diagnosis*.

[34] Qureshi I. A., Ullah H., Akram M. H., Ashfaq S., Nayyar S. (2004). Transvaginal versus transabdominal sonography in the evaluation of pelvic pathology. *Journal of the College of Physicians and Surgeons--pakistan: JCPSP*.

[35] Coleman B. G. (1992). Transvaginal sonography of adnexal masses. *Radiologic Clinics of North America*.

[36] Baschat A. A., Gembruch U. (1998). Ante- and intrapartum diagnosis of vasa praevia in singleton pregnancies by colour coded doppler sonography. *European Journal of Obstetrics & Gynecology and Reproductive Biology*.

[37] Catanzarite V., Maida C., Thomas W., Mendoza A., Stanco L., Piacquadio K. M. (2001). Prenatal sonographic diagnosis of vasa previa: ultrasound findings and obstetric outcome in ten cases. *Ultrasound in Obstetrics and Gynecology*.

